# The Effect of Nursing Intervention on Patients with Inguinal Hernia and Its Influence on Self-Management Ability

**DOI:** 10.1155/2022/4965709

**Published:** 2022-08-05

**Authors:** Ning Zhang, Jingjing Miao, Qiaona Zheng

**Affiliations:** General Surgery of Funan County People's Hospital, Fuyang, China

## Abstract

**Objective:**

To objectively evaluate the nursing quality of patients with inguinal hernia from the aspects of postoperative pain, self-discipline, and complications, the application of medical data analysis and nursing intervention in patients with inguinal hernia was discussed.

**Methods:**

A total of 86 patients with inguinal hernia were selected, and the time distribution was from September 2020 to March 2021. The patients were divided into two groups: in the control group, there were 43 cases, 28 males and 15 females. There were 43 cases in the observation group, 25 males and 18 females. All selected subjects must sign the informed consent form and have the right to know the research content. The patients were diagnosed by abdominal ultrasound, and the demographic data and basic clinical data were recorded.

**Results:**

A total of 86 patients were divided into two groups in this study, of which 43 patients used a routine nursing path as the control group and the other 43 patients added medical data analysis and nursing intervention as the observation group on the basis of the routine nursing path. The postoperative pain, self-discipline, complications, and patient satisfaction were compared, and the patients' satisfaction in the experimental group was significantly higher than that in the control group, while serum swelling and urine retention were significantly lower than those in the control group (*p* < 0.05).

**Conclusion:**

According to the analysis of the routine nursing path and medical data, nursing intervention patients have more stable emotions and less postoperative pain. They can get out of bed early, reduce the occurrence of other complications, and improve the overall curative effect. Systematic nursing intervention can reduce the incidence of postoperative adverse reactions and complications. It is one of the ideal adjuvant treatments for inguinal hernia patients.

## 1. Introduction

An inguinal hernia is a common surgical disease from infants to the elderly, regardless of age [1]. The cause is often related to family genetic history, age, and gender. The decrease in abdominal diaphragm muscle strength and the increase in intraperitoneal pressure are the main causes of abdominal wall hernias. The clinical symptoms are often manifested as a prominent mass in the groin. When people stand up and do heavy physical labor, an obvious mass can be seen by the naked eye in the groin. When sleeping, the mass can disappear with the decrease in intraperitoneal pressure.

Hernias can be understood as the displacement of internal organs and tissues formed when the internal organs and tissues of the human body leave the original position [2]. An inguinal hernia is located in the lower triangular area of the human abdomen, which is connected with the inguinal ligament and rectus abdominis. For inguinal hernia surgery, one-time surgical treatment can be used, with the help of surgical measures to repair the hernia, and the postoperative recurrence is small. If conservative treatment is adopted, antibiotics need to be taken for a long period of time.

With the help of physical therapy, infants and young children have a certain chance to recover from abdominal hernia by themselves. The elderly and infirm can also intervene through physical methods and take drugs to reduce the occurrence of inflammation. Other patients usually recommend surgical treatment to avoid constipation and physical labor. In the case of increased abdominal pressure such as coughing or sneezing, the intestines and spermatic cords may break through the weak parts of the groin, which will increase the abdominal pressure, promote weight gain, affect the injury of abdominal wall muscles, aggravate the pain of patients, and also lead to the secondary recurrence of inguinal hernia, and even endanger their lives in serious cases [3]. According to the actual situation of patients, most patients with inguinal hernia are treated by using a surgical suture or patch repair, but however, whether suture technology or patch repair technology, there will be a chance to increase the risk of infection for patients. Patients will face the possibility of long hospital stay, high medical costs, recurrence, and deterioration of their condition. At the same time, it will also increase the potential risk of intestinal fistula, intra-abdominal abscess, and huge incisional hernia [4].

Now, big data is increasingly used in medicine. Combined with the application of medical data analysis in postoperative nursing, targeted nursing can be carried out according to the situation of patients, making the application of nursing more specific. It can not only improve the quality of life of patients after operation but also reduce the occurrence of other complications. Hanna's scientific nursing intervention can help improve the symptom self-assessment of patients with inguinal hernia after tension-free repair, reduce their stress state, meet their nursing needs, improve their safety, and then promote their rehabilitation [5]. This study analyzed the whole process of postoperative nursing intervention for patients with an inguinal hernia and clarified the role of medical data in postoperative nursing intervention for patients with an inguinal hernia.

## 2. Literature Review

Excessive exercise or heavy physical labor can increase abdominal pressure, resulting in the displacement of abdominal organs and the formation of hernias. Using surgery to solve the inguinal hernia caused by trauma is the most common method, and the trauma surface is small and not easy to relapse.

Surgery has a certain risk of infection and complications. Combined with the fusion of medical data, we can strengthen the intervention of nursing means in the postoperative situation of patients so as to reduce the pain of patients, alleviate their emotional discomfort, contribute to the recovery of the disease, and improve the curative effect.

There are certain risks in any surgical operation, and especially, the surgical scheme of inserting foreign bodies into the body makes the risk of infection rise sharply. In this paper, the method of patch repair is used to repair the muscle weakness of inguinal hernias in the elderly and to explore the effect of high-quality nursing in the process of postoperative intervention. Finally, it is concluded that the application of high-quality nursing in the postoperative repair of inguinal hernia muscle weakness in the elderly can improve the postoperative recovery effect of patients and reduce the risk of other complications [6]. Children are prone to inguinal hernias. Crying or emotions will increase the swelling of an abdominal hernia mass and affect their condition. In this paper, the application of comfort nursing for children after inguinal hernia repair was introduced, and the effect was observed. A total of 118 pediatric patients were selected for follow-up. Finally, it was found that the pediatric patients with comfortable nursing had stable emotion and less pain and discomfort, which was helpful to their physical recovery and reduced the occurrence of postoperative complications [7].

Clinical surgical measures can only solve the serious illness of patients and the body but cannot eradicate the psychological panic of patients. Postoperative nursing intervention can give emotional comfort so as to reduce psychological discomfort. In this paper, the high-quality nursing was involved in the whole process of service for patients with indirect inguinal hernias after operation, and the changes in patients' psychology, pain, and emotion were explored. Through experimental comparison, it is finally concluded that high-quality nursing can improve patients' anxiety and relieve tension so as to reduce postoperative pain, and a positive attitude is conducive to the recovery of the disease [8]. This method can reduce the pressure of abdominal hernias and increase the effect of abdominal hernia repair through the intervention of Liu Zhongtian tablet [9].

Although the nursing intervention method combined with medical data is less effective than the direct effect of clinical surgery on patients' conditions, its effect cannot be ignored. Relevant data show that nursing intervention can improve the success rate of surgery, reduce postoperative complications, calm patients' emotions, and guide patients to transfer psychological anxiety with a positive attitude [10].

Mengya clinical medicine usually uses the patch to repair the abdominal diaphragm to treat an inguinal hernia. This paper analyzes the whole process of the nursing intervention value of patients after operation. Through comparison, the patients with whole course nursing intervention get out of bed earlier than those with routine nursing, and the abdominal incision pain is less, which can promote the recovery of patients as a whole [11].

## 3. Data and Methods

### 3.1. Object Selection

Eighty-six patients with inguinal hernias hospitalized in our hospital from September 2020 to March 2021 were divided into two groups. 43 cases in the control group, 28 males and 15 females, aged (16–86) years, with an average of (46.23 ± 7.63) years. There were 43 cases in the observation group, 25 males and 18 females, aged (15–79) years, with an average of (53.44 ± 8.91) years. All selected subjects need to sign the informed consent form and have the right to know the contents of the study.

### 3.2. Inclusion Criteria

Patients with inguinal hernia disease diagnosed by ultrasound and other methods and suitable for surgical treatment should seek medical examination in time after onset and meet the standards of hospitalization.

Patients with other diseases, such as patients with malignant tumors or serious lesions of other organs, those with a history of open abdominal surgery and no civil capacity, those with incomplete clinical data, those who refuse to cooperate, or those who are not suitable for participating in the investigation for other reasons, are excluded. All patients participating in the investigation in this study have the right to know.

### 3.3. Grouping Method

Control group: a routine nursing path was used which involved communicating with patients and their families before operation, soothing patients' preoperative psychology, alleviating patients' perioperative psychological anxiety, and counseling patients with psychological problems. It also has the obligation to inform patients and their families of perioperative precautions, give guiding intervention to patients' postoperative rehabilitation, and improve patients' and their families' postoperative cooperation and compliance.

Observation group: nursing intervention based on medical data analysis was used. Combined with the basic data of clinical medicine, life and health-related data, and hospital infrastructure, through the statistics and analysis of intelligent data analysis tools, the hospital can apply the analyzed data to nursing and then conduct a more detailed evaluation of patients after nursing in combination with the conventional nursing path.

### 3.4. Observation Index

(1) Operation indexes: the visual analogue pain (VAS) scale was used to evaluate the pain of patients in the two groups on 1D, 2D, 3D, 4D, and 5D after operation (a total of 10 points). (2) Patients' self-restraint ability: the two groups of patients with abdominal hernias were evaluated by a self-restraint ability questionnaire before and after nursing from five aspects: general state analysis, psychological behavior, diet, problem handling, and emotional expression. The total score was 20 points. The higher the score, the stronger the self-restraint ability. (3) Postoperative complications and the right to know: the incidence of postoperative serum swelling and urinary retention in two groups of patients with abdominal wall hernias was recorded. After nursing, the two groups were evaluated by the questionnaire from the causes of disease, treatment plan, and exercise recovery. The total score of each item was 100, and the awareness rate was ≥90.

### 3.5. Statistical Methods

SPSS data analysis was used to explore the effect of medical data analysis and nursing intervention in patients with inguinal hernias.

The statistical method for determining the value of coefficient R2 is shown in the following formula:

(1) $$\begin{array}{c} R^{2}=\frac{\sum_{i}\left(x_{i}-\bar{x}\right)}{\sum_{i}\left(x_{i}-{\tilde{x}}_{i}\right)},\;\bar{x}=\frac{1}{n}\sum_{i=1}^{n}x_{i}. \end{array}$$

Here, $\bar{x}：$ input the sequence to calculate the average value, ${\tilde{x}}_{i}$ is the ith input data, *x*_*i*_is the ith input data, and *n* is the sample maximum subscript.

The calculation algorithm of the *T* value (value) is shown in the following formula:

(2) $$\begin{array}{c} t_{\text{Value}}=\frac{\left(\bar{x}-\mu \right)}{\sigma_{x}/\sqrt{n-1}},\bar{x},\mu \\ =\frac{1}{n,m}\sum_{i=1}^{n,m}x_{i},\sigma_{x}\\ =\frac{1}{\left(n-1\right)}\sqrt{\sum_{i=1}^{n}{\left(x_{i}-\bar{x}\right)}^{2}}. \end{array}$$

Here, $\bar{x}$ is the mean value, *μ* is the reference mean value, n is the sample maximum subscript, m is the maximum subscript of the reference sample, and *σ*_*x*_ is the sample standard deviation.

## 4. Results

### 4.1. Comparison of the Pain Degree between the Two Groups in Different Nursing Interventions after Operation

The pain rating scale (VAS) evaluates postoperative nursing pain perception from the perspective of patients' subjective evaluation. The score is divided into four levels, ranging from 0 to 10. According to the degree of pain, 0 is the lowest and 10 is the highest. The scores of all patients were statistically analyzed. The data obtained are shown in Table 1.

In Table 1, the pain perception evaluation of patients with inguinal hernias in the two groups from 1 to 4 days after operation was statistically significant (*p* < 0.05), while the pain data of patients in the five days after operation were not statistically significant, indicating that after intervention with different nursing methods, the pain of patients in the observation group was lower than that in the control group, indicating that the nursing methods in this study can reduce the pain of patients to a certain extent and make patients feel more comfortable in the process of rehabilitation, and it is helpful for the postoperative recovery of patients. According to the evaluation results in Table 1, it is transformed into a visual diagram, as shown in Figure 1.

As can be seen more clearly from Figure 1, after nursing, the pain of patients in both groups was relieved. The pain of patients with inguinal hernias in the observation group is much lower than that of patients in the control group. Compared with the scores of patients with inguinal hernias in the control group, the observation group has more advantages, which shows that the nursing intervention based on medical data analysis proposed in this study is more scientific and conducive to the postoperative rehabilitation of patients with inguinal hernias.

### 4.2. Comparison of the Postoperative Restraint Behavior between the Two Groups of Patients with Inguinal Hernias

A questionnaire survey was designed for the general state management, social psychological behavior, diet management, problem solving, and emotional treatment of inguinal hernia patients with different nursing interventions before and after nursing. All patients were scored. The evaluation data were statistically analyzed. The data obtained are detailed in Table 2.

In Table 2, there was a significant difference in the self-restraint behavior between the two groups before nursing compared with that before treatment (*p* > 0.05). The score of the self-restraint behavior ability of patients with inguinal hernias after nursing was higher than that before nursing (*p* < 0.05). The observation group had certain advantages in general state management, social psychological behavior, diet management, problem solving, and emotional therapy. According to the data in the above table, Figure 2 can more clearly show the comparison of the self-restraint behavior ability of inguinal hernia patients with different nursing interventions.

In Figure 2, the five indexes of the self-restraint behavior ability of patients in the control group after routine nursing are lower than those of patients intervened by nursing means based on medical data analysis, which shows that the nursing path through targeted data analysis is more in line with the current situation of patients. Therefore, the evaluation of self-restraint behavior ability indexes such as overall situation, psychological behavior, and diet management has certain advantages.

### 4.3. Comparison of Postoperative Complications and the Awareness Rate between the Two Groups of Patients with Inguinal Hernias

The patients with inguinal hernias after different nursing interventions were followed up, and the postoperative complications of all patients and the awareness rate of the condition were statistically analyzed, as shown in Table 3.

In Table 3, after 22^*∗*^*T* check (*p* < 0.05), the incidence of serum swelling and urinary retention in the observation group was relatively low, and the control group had a higher awareness rate of pathogenesis, treatment, and rehabilitation exercise. This also shows that after the nursing intervention based on medical data analysis, the risk rate of other accompanying symptoms in patients with inguinal hernias is much lower than that in patients with routine nursing in the control group. In order to more intuitively reflect the analysis and comparison results of the risk rate of other accompanying symptoms of inguinal hernia patients and the risk rate of routine nursing patients in the control group after the nursing intervention based on medical data analysis, the comparison results of postoperative complications and awareness rate of the two groups in Table 3 are visualized, and Figure 3 is obtained:

In Figure 3, the risk of postoperative serum sore-associated symptoms in patients with inguinal hernias after medical data analysis is 0%, and the probability of occurrence of urinary retention is 2.33%, which is significantly lower than that of the control group. The awareness rate of the pathogenesis, treatment methods, and rehabilitation exercise of the disease is also much higher than that of the patients in the control group, which shows that the patients in the observation group pay more attention to their physical recovery after nursing than that of the control group.

### 4.4. Comparison of Postoperative Nursing Service Satisfaction between the Two Groups

In order to evaluate and verify the effect and practical value of the nursing intervention for inguinal hernia patients based on medical data analysis proposed in this study, a questionnaire survey was made to let these patients evaluate the nursing quality and personnel satisfaction. The specific data are shown in Table 4.

In Table 4, the patients in the observation group were 97.57% satisfied with the quality of care given by the hospital according to the analysis of medical data, and 98.41% were satisfied with the service attitude of nursing staff. The patients in the control group were 73.94% satisfied with the quality of nursing and 75.97% satisfied with the service attitude of nursing staff. From these data, it can be seen that the patients in the observation group were more satisfied with the quality of nursing and the service attitude of nursing staff than those in the control group.  Figure 4 is obtained according to the evaluation data of patients' satisfaction with nursing.

In Figure 4, it can be seen that the data of the observation group are better than those of the control group in terms of satisfaction evaluation of the nursing quality and nursing service attitude, which shows that the method proposed in this study is more acceptable and loved by patients with inguinal hernias than conventional nursing.

## 5. Discussion

An inguinal hernia is a common surgical disease. Its pathogenesis is not clear. It often occurs in people of all ages, and it is one of the most common diseases in surgery. It mainly destroys the abdominal tendons, pressing the internal organs of the abdomen to move to the weak area of the abdominal wall, which leads to organ displacement. Surgical repair of the abdominal diaphragms is commonly used in clinics. However, patch repair technology also has many postoperative problems. The infection, organ damage, and other problems it bring will make chronic pain increase day by day. The placement of patches in the body also greatly increases the risk of abdominal infection, which will bring a certain burden to the patient's psychology, resulting in poor postoperative cooperation and affecting the postoperative curative effect.

This study is combined with medical data to carry out nursing intervention on patients and carried out machine learning analysis on the data of patients' vital signs and hospital basic facilities so as to finally get the best nursing path and carry out targeted nursing intervention on patients after operation. The pain, postoperative self-restraint, postoperative complications, and the right to know were evaluated. The nursing quality of patients was evaluated by a questionnaire. The nursing intervention of medical data blindly adopts the means of emotional comfort compared with conventional nursing methods, which is more targeted. It can substantially solve the needs of patients, fundamentally alleviate the pain of patients, stabilize the emotion of patients, eliminate emotional discomfort, and contribute to the recovery of the disease.

Yang mentioned in the application analysis of comprehensive nursing intervention in patients undergoing laparoscopic inguinal hernia repair that the treatment effect of the abdominal hernia using a patch is not only directly related to surgical measures but also indirectly related to perioperative nursing intervention. Combined with scientific nursing intervention methods, it can strengthen the surgical effect, improve patients' psychological anxiety, and reduce the incidence of postoperative complications [12]. Because children are young, their mental development is not perfect and they have psychological fear of clinical surgery. According to this characteristic, this paper increases clinical nursing work to intervene in psychological intervention during surgery for children with inguinal hernias so as to reduce the negative impact of emotional pressure on the condition [13]. Clinical medicine usually uses the patch to repair the abdominal diaphragm to treat inguinal hernias. This paper analyzes the whole process of the nursing intervention value of patients after operation. Through comparison, the patients with the whole course nursing intervention get out of bed earlier than those with routine nursing, and the abdominal incision pain is less, which can promote the recovery of patients as a whole.

All investigators need to sign informed consent. The relevant medical data of patients belong to the privacy of patients. All examination results and privacy of patients are protected and shall not be published. Without violating the confidentiality principle and relevant laws and regulations, only the personnel participating in the study can access the basic clinical data of patients.

## 6. Summary

The curative effect of abdominal hernia repair is not only directly related to surgical measures but also indirectly related to perioperative nursing intervention. Appropriate nursing should be used during the operation; otherwise, it is easy to have adverse reactions and affect the quality of life of patients. Nursing intervention in the whole course of treatment can not only improve clinical symptoms but also improve the clinical effect, prognosis, and quality of life of patients. Combined with scientific nursing intervention, it can enhance the effect of operation, improve the psychological anxiety of patients, and reduce the occurrence of postoperative complications, and it can effectively improve the nursing satisfaction rate of patients. Through the grouping experiment, the postoperative pain, self-control, complications, and patient satisfaction were compared. From the perspective of postoperative patients' psychological impact, emotional fluctuation, and infection risk, the emotion of patients with the whole course nursing intervention is more stable than that of patients with routine nursing so as to reduce patients' complications and improve the treatment effect. Nursing intervention is an auxiliary means of treatment and plays a positive role in the treatment of patients. There is still a broad space for development in this field to help patients with postoperative rehabilitation.

## Figures and Tables

**Figure 1:** Comparison of the VAS score data after operation between the two groups.

**Figure 2:** Comparison of the self-restraint behavior ability between the two groups of patients with inguinal hernias after nursing.

**Figure 3:** Comparison of postoperative complications and the awareness rate between the two groups.

**Figure 4:** Comparison of postoperative nursing satisfaction evaluation between the two groups.

**Table 1:** Comparison of postoperative VAS scores of patients with inguinal hernias between the two groups $\left(\bar{x}\pm s\right)$.

Group	Number	1 day	2 days	3 days	4 days	5 days
Observation group	43	6.16 ± 0.52	4.32 ± 0.35	3.02 ± 0.21	1.57 ± 0.21	1.02 ± 0.31
Control group	43	7.91 ± 0.61	6.48 ± 0.43	4.05 ± 0.36	2.85 ± 0.35	1.05 ± 0.33
t	—	5.337	5.268	5.104	5.197	0.172
*p*	—	0.008	0.005	0.004	0.006	0.341

**Table 2:** Performance of self-restraint behavior ability of patients with inguinal hernias in the two groups before and after nursing $\left(\bar{x}\pm s\right)$.

Group		General status management	Psychosocial behavior	Diet management	Problem solving	Emotional processing
Observation group (*n* = 43)	Before nursing	11.29 ± 1.73	12.51 ± 1.78	11.57 ± 1.76	12.01 ± 2.15	11.99 ± 1.79
	After nursing	17.43 ± 1.98^#*∗*^	18.43 ± 1.53^#*∗*^	16.78 ± 1.67^#*∗*^	18.21 ± 1.74^#*∗*^	17.93 ± 1.95^#*∗*^

Control group (*n* = 43)	Before nursing	11.31 ± 1.75	12.53 ± 1.80	11.61 ± 1.79	12.04 ± 2.17	12.00 ± 1.82
	After nursing	14.69 ± 1.84^*∗*^	15.31 ± 1.69^*∗*^	14.21 ± 1.69^*∗*^	15.32 ± 1.93^*∗*^	14.69 ± 1.89^*∗*^

**Table 3:** Comparison of postoperative complications and awareness rate between the two groups (*n*(%)).

Group	Number of cases	Postoperative complications			Awareness rate		
		Seroma	Uroschesis	Incidence rate	Pathogenesis	Therapeutic method	Rehabilitation exercise
Observation group	43	0(0.00)	1(2.33)	1(2.33)	41(95.35)	42(97.67)	43(100.00)
Control group	43	2(4.65)	4(9.30)	6(13.95)	35(81.40)	37(86.05)	39(90.76)
*x* ^2^	—	1.367	3.249	3.888	4.074	3.888	4.195
*p*	—	0.001	0.045	0.049	0.044	0.049	0.041

**Table 4:** Evaluation of postoperative nursing satisfaction of patients with inguinal hernias in the two groups.

Group	Number of cases	Service quality satisfaction	Satisfaction rate of medical staff	Comprehensive satisfaction
Observation group	43	97.57%	98.41%	97.28%
Control group	43	73.94%	75.97%	74.29%
t	—	1.364	1.427	1.367
*p*	—	0.006	0.004	0.003

## Data Availability

The data underlying the results presented in the study are included within the manuscript.
